# The Design, Fabrication and Characterization of Grating Couplers for SiGe Photonic Integration Employing a Reflective Back Mirror

This article has been retracted.

**DOI:** 10.3390/nano12213789

**Published:** 2022-10-27

**Authors:** Qiang Huang, Yi Zhang, Jie Tang, Junqiang Sun

**Affiliations:** 1 Hunan Provincial Key Laboratory of Grids Operation and Control on Multi-Power Sources Area, School of Electrical Engineering, Shaoyang University, Shaoyang 422000, China; jie_syust@126.com; 2 Wuhan National Laboratory for Optoelectronics, School of Optical and Electronic Information, Huazhong University of Science and Technology, Wuhan 430074, China; yihust@163.com (Y.Z.); dbhust@126.com (J.S.)

**Keywords:** silicon photonics, SiGe modulator, vertical coupling, grating coupler, metal reflective layer

## Abstract

We propose and demonstrate an efficient grating coupler for integrated SiGe photonic devices. A bottom metal layer is adopted to enhance the coupling efficiency on the wafer backside. A low coupling loss of −1.34 dB and −0.79 dB can be theoretically obtained with optimal parameters for uniform and apodized grating couplers, respectively. The fabrication process is CMOS compatible without need of wafer bonding. The influence of fabrication errors on the coupling efficiency is analyzed in terms of substrate thickness, grating dimension and material refractive index. The results indicate a large tolerance for the deviations in practical fabrication. The measured coupling loss of the uniform grating is −2.7 dB at approximately 1465 nm with a 3 dB bandwidth of more than 40 nm. The proposed grating coupler provides a promising approach to realize efficient chip-fiber coupling for the SiGe photonic integration.

## 1. Introduction

In the past few years, there has been extensive progress in silicon photonics [1,2,3]. The SiGe material platform is considered as a promising solution to achieve highly efficient active and passive intergraded devices with the complementary metal-oxide semiconductor (CMOS) technology. Although Ge is an indirect bandgap semiconductor, the indirect L-valley band edge is only approximately 140 meV lower than the direct Γ-valley band edge and the direct bandgap optical properties of Ge have been heavily explored [4,5,6]. In recent years, Ge/SiGe quantum wells have been intensively studied [7,8,9] and much progress has been made for the optical modulators, photodetectors and emitters within the communication wavelength in silicon-based integrated optoelectronic devices [10,11,12,13].

Numerous on-chip devices eventually need to couple light from or to optical fibers. However, there are few reports about the grating couplers developed in the integrated SiGe semiconductor devices. Most works are using the butt-coupling scheme for transferring the optical power from the single mode fiber (SMF) to the SiGe waveguide. This usually leads to quite a few coupling losses since it is difficult to fabricate SiGe waveguides with high quality facets [14]. As an alternative approach for coupling light from or to the submicron-sized waveguide, the surface grating coupler has inherent advantages over the edge coupler. The grating coupler can be placed anywhere on the chip surface and does not require polishing of facets, which increases design flexibility and enables wafer scale optical testing in mass production. It also has a large tolerance for spatial alignment due to vertical coupling. In addition, the grating coupler can be realized as one or two-dimensional structures and can help to couple one or both orthogonal polarization states, acting as polarization beam splitters [15,16]. Many significant breakthroughs have been made for the grating couplers of the silicon-on-insulator (SOI) platform [17,18,19,20], but fiber-chip coupling is still a big challenge for SiGe semiconductor devices. It is noticed that some achievements have been made for the Ge grating couplers, but the results are not so impressive and they are all designed for the mid-infrared (mid-IR) applications [21,22,23]. Thus, it is necessary to investigate and design an efficient grating coupler for the SiGe photonic integration.

In this paper, we propose and demonstrate an efficient grating coupler for the integrated SiGe waveguide on Si substrate. In order to obtain a high coupling efficiency, a bottom metal layer is employed on the wafer backside to reflect back downward optical power. By carefully optimizing the groove width, the grating period and etch depth of the grating coupler, a high coupling efficiency of −1.34 dB and −0.79 dB can be theoretically acquired for the uniform and non-uniform SiGe grating couplers, respectively. The deviations in the practical production are discussed in detail and the proposed grating coupler shows satisfactory robustness for the fabrication errors. The measured coupling loss is −2.7 dB at approximately 1465 nm with a 3 dB bandwidth of more than 40 nm. Simulated and experimental results both signify that the designed grating coupler can be a promising candidate for efficient chip-fiber couplers in the integrated SiGe photonic devices.

## 2. Design and Simulation

The structure of the proposed grating coupler is shown in Figure 1. A Ge_0.85_Si_0.15_ layer that is 1 μm thick is deposited on Si substrate and the grating coupler is covered by a SiO_2_ cladding layer, which is optimized to not only protect the whole device but to also enhance the coupling efficiency. Unlike the SOI platform, the refractive index difference between SiGe waveguide and Si substrate is too small, so the majority of light coupling from the single mode fiber diffracts to the substrate. In order to achieve a high coupling efficiency, a bottom metal layer is adopted as a perfect mirror to reflect back downward optical power. For the convenience of fabrication, the windows of the metal mirrors are defined on the wafer backside and are wet or dry etched until the Si substrate is only several microns thick. Then, an appropriate metal (e.g., aluminum) layer is deposited in the etch trench by electron beam evaporation. This cost-effective procedure is CMOS compatible [24] and much simpler than the wafer bonding process that is utilized for the bottom distributed Bragg reflector structure [25].

First of all, the designs for grating couplers should be satisfied with the Bragg condition, which can be expressed as

(1) $$k_{in}\sin\theta +mk_{gc}=\beta ,\;m=\pm 1,\pm 2,\cdots$$

where *k_in_* = 2*πn_c_*/*λ*_0_ is the incident wave number with the refractive index of the top cladding layer *n_c_* and the free space wavelength *λ*_0_, *θ* is the fiber off-vertical tilt angle, *m* is the diffraction order, *k_gc_* = 2*π*/*p* is the grating vector with the grating period *p*, and *β* = 2*πn_eff_*/*λ*_0_ is the propagation constant of the optical mode in the gratings with the effective refractive index *n_eff_*. Generally, it is expected to have a maximum coupling efficiency only for the diffraction order *m* = 1.

The optimizations are investigated using a commercial 2D finite-difference time-domain (FDTD) numerical simulation tool with a grid size of 20 nm, which is produced by Lumerical Solutions. A Gaussian source with a mode field diameter of 10.4 μm is employed to represent the single mode fiber input. The optimized fiber off-vertical tilt angle of *θ* = 9° is adopted to avoid the second-order reflection. The coupling efficiency is defined as the ratio of detected power in the fundamental mode at the waveguide to the input power, and the coupling efficiency can directly reflect the loss of the grating region because the loss of the grating region is significantly larger than that of the angle-optimized taper. Since the operation wavelength of SiGe/Ge multiple quantum wells is usually at the short wavelength band (S-band) and extended wavelength band (E-band) of optical communication [26,27], the proposed grating coupler is designed for the corresponding band and optimized for transverse electric (TE) mode.

For the common uniform grating couplers, the coupling efficiency depends on the groove width *w*, the grating period *p* and the etch depth *h*. Usually, the etch depth has a more significant influence on the effective refractive index of gratings than the groove width and the grating period. On one hand, the etch depth should not be too large to avoid the back reflection at the interface between the waveguide and the grating region. On the other hand, it should not be too small to maintain enough coupling strength of the gratings. So, the coupling efficiency is more sensitive to the etch depth than the other two parameters and a relatively high coupling efficiency can be obtained in a large range of the groove width and grating period for a given etch depth of grating couplers. Therefore, the influence of etch depth of the grating is first assessed at the Si-substrate thickness of 2 μm, the grating period of 780 nm and the groove width of 400 nm with a SiO_2_ cladding layer that is 100 nm thick. The period number of the grating is set to 18, which is obtained by the simulation scan, and the input position is adjusted to maximize the coupling efficiency.

Then, we scan the wavelength with 1 nm steps in the 1420 nm to 1500 nm range, and we scan the etch depth with 10 nm steps in the 300 nm to 450 nm range. Figure 2 illustrates the calculated coupling efficiency as a function of the etch depth and operation wavelength. It can be observed that the highest coupling efficiency of 75% is obtained with the etch depth *h* = 370 nm at the wavelength of 1470 nm. Considering the 3 dB bandwidth and the fabrication deviations, the optimal etch depth *h* = 380 nm is chosen with the highest coupling efficiency of 73% at 1466 nm.

After fixing the best etch depth of the grating couplers, the groove width and grating period are optimized similarly. Finally, the etch depth *h* of 380 nm, the grating period *p* of 780 nm and the groove width *w* of 400 nm are chosen as the optimal parameters for the gratings. Figure 3 implies the calculated coupling efficiency spectra of the proposed structure with and without the metal mirror. It can be seen that a coupling efficiency of −1.34 dB is acquired at 1466 nm with the metal layer, which is remarkably ameliorated from −10.73 dB at 1460 nm without the metal layer. Since the diffracted optical power toward the substrate is reflected back at the metal mirror, a large portion of light is redirected to the waveguide output and the coupling efficiency of the grating coupler is improved by approximately 9.4 dB. The 3 dB-bandwidth of 36 nm is obtained, which is smaller than the Si grating coupler of the SOI platform. This is mainly due to the higher effective refractive index and thicker waveguide of the SiGe grating coupler.

Figure 4 shows the simulated electrical field component *E_Z_* distribution and optical power distribution of the grating coupler with and without the metal mirror. It turns out that the grating directionality improves enormously and the output optical field is well restricted in the waveguide with the metal mirror underneath. Due to the reflection of the bottom metal mirror, the power superposition is different at different positions. Thus, there is a vertical shift in the optical power distribution toward the end on the grating in Figure 4b. Additionally, the horizontal line in Figure 4 represents the main area of light field propagation.

For a uniform grating, the diffracted field profile is exponentially decaying along the propagation direction of the grating structure and there is a considerable mismatch with the Gaussian field profile of the optical fiber. The coupling efficiency can be further enhanced by increasing the field overlap between the fiber and grating coupler with a non-uniform structure [28,29]. In order to realize a near-Gaussian diffracted field, an apodized grating coupler is explored by varying the groove width and grating period, while keeping the etch depth constant for a single etch step. On the SOI material platform, the effect of two-step apodization grating in improving the mode matching is close to that of the continuous apodization, which is demonstrated by the state of the art [30]. Thus, we use the two-step apodization scheme to enhance the coupling efficiency, which can avoid complex genetic algorithms to optimize the structure of continuous apodization and simplify the fabrication process. The two-step apodized grating consists of two grating sections, the first part consists of four grating periods with the groove width of 100 nm and the period of 690 nm, followed by 14 periods with the groove width of 400 nm and the period of 780 nm as the second section. The minimum feature size is compatible with the current deep ultraviolet (DUV) lithography, which enables large volume fabrication at a low cost. Figure 5 indicates the calculated coupling efficiency as a function of wavelength for the uniform and the apodized grating coupler. The highest coupling efficiency of −0.79 dB is achieved at 1466 nm with a 3 dB-bandwidth of 36nm for the apodized design, exhibiting an appreciable improvement of 0.55 dB in comparison with the uniform grating coupler.

## 3. Tolerance Analysis

In the practical material growth and fabrication of the grating coupler, there are always some deviations from the desired grating structure. These deviations have an impact on the coupling efficiency due to the variations in resonance wavelength, coupling strength and effective refractive index. Thus, it is necessary to evaluate the tolerance of the proposed grating coupler for fabrication errors. Similar results can be obtained when considering the apodized grating, hence we only display the discussion about the uniform grating coupler here.

One of the fabrication errors is the thickness of the Si substrate between the metal layer and the SiGe waveguide. We set the thickness to 2 μm in the aforementioned design, but it is difficult to control the thickness precisely in the actual etching process [31]. The thickness is investigated since it can produce the interference effect between the diffracted field toward the waveguide layer and the field that is reflected at the bottom metal mirror. Figure 6 shows the simulated coupling efficiency of the coupler as a function of the substrate thickness after etching at the wavelength of 1466 nm. It can be apparently observed that the coupling efficiency periodically depends on the thickness and the constructive interference occurs at the peak point while the destructive interference occurs at the valley point. The thickness range corresponding to 3 dB and 1 dB declining in the coupling efficiency is, respectively, approximately 163 nm and 125 nm, which is enough to afford the fabrication errors of etching depth.

Owing to the proximity effects in the DUV lithography, it is inevitable to cause the deviations with respect to the expected dimension of the grating coupler. Here, we focus on the variations of the groove width *w* since the grating period usually remains unchanged. Figure 7 indicates the calculated coupling efficiency spectra in reference to the groove width variation Δ*w*. It can be seen that the resonant wavelength has a small blue shift and the 3 dB bandwidth decreases slightly with the increasing groove width. In the case of decreasing groove width, the highest coupling efficiency declines mildly, but the 3dB bandwidth has a modest enhancement. Considering the typical dimensional control range within 10 nm in photonic foundries [32], the proposed grating coupler still has a strong fabrication tolerance for the dimension deviations.

Limited by the material growth technology, the instability of vapor deposition processes generally introduces a deviation of Ge composition varying from −2% to 4% [33], which results in a refractive index variation of approximately ±0.03 for the SiGe alloy. Figure 8 shows the simulated coupling efficiency as a function of wavelength for different refractive index variation Δn. It is clear that the increment of refractive index leads to a slight red shift of the resonant wavelength, while the case of decrement of refractive index is just opposite. The highest coupling efficiency for both variations is close to the desired design and the difference is within the acceptable range.

## 4. Fabrication and Measurement Results

Figure 9 depicts the fabrication process of the whole device. The grating and waveguide are both patterned by the electron beam lithography (EBL) and etched by the inductively coupled plasma (ICP) etcher to ensure high accuracy. Then, the device is covered by a layer of SiO_2_ passive cladding. Next, we turn over the chip and define the windows of metal layers on the chip backside with a double-faced lithography machine. The double-faced lithography machine with the backside alignment accuracy of 500 nm is MA8. Then, we deeply etched the widow. However, long time etching will cause overheating of the equipment, and a signal ICP etching time should not exceed two hours. Two hours of deep etching could not reach the required depth, thus, we then performed wet etching at a temperature of 80 °C using a solution diluted with 25% tetramethylammonium hydroxide (TMAH) and deionized water at a volume ratio of 1:4.

Finally, the windows are deeply etched, followed by the 10 nm/100 nm Cr/Au metal layer lithography, evaporation and lift-off. Figure 10 shows the SEM images of the uniform grating and metalloscope images of the metal layers on the chip backside. The etch depth of the fabricated uniform grating is approximately 385 nm and the period is 779.5 nm with the groove width of 404.3 nm, which are close to the designed dimensions. The etch depth and width of the waveguide are 640 nm and 2 μm, respectively, and the height of the SiGe cladding is 100 nm. Several waveguides of different length are simultaneously fabricated to evaluate the optical propagation loss for accurate measurements of the coupling loss. The length and width of the tapers are 100 μm and 15 μm, respectively, and the angle of the taper is 23° consistent with the simulation optimization results. Additionally, the optical spot converting loss is below 0.22 dB for each side taper. As can be seen from Figure 10c,d, the backside of the chip is rough since it is not polished. To decrease the roughness of the metal layer, the diluent TMAH solution is employed to smoothen the surface of the deeply etched trench before metal evaporation.

We use a pair of single mode fibers to couple light into and from the SiGe gratings, and the test setup is shown in Figure 11. The light from a tunable laser is first injected into a polarization controller to obtain a transverse electric field input. The output light emerging from the grating is detected by an optical power meter. To ensure the highest coupling efficiency, we employ a set of precision optical fiber regulating frames to adjust the position of the fibers until the output optical power is maximal. Figure 12 illustrates the coupling efficiency of the uniform grating as a function of the wavelength for TE mode. The measured highest coupling efficiency is −2.7 dB at approximately 1465 nm, which is lower than the simulated coupling efficiency of −1.34 dB at 1466 nm. The additional coupling loss might be because of the scattering loss from the metal layer since the bottom etched trench is not smooth enough. The 3 dB bandwidth of the fabricated grating is more than 40 nm, even though the measurement range is limited by the wavelength range of our tunable laser. We also make measurements for the same grating without a metal layer, but no obvious transmission of light is observed.

## 5. Conclusions

In summary, we have proposed and demonstrated an efficient grating coupler with a bottom metal layer for SiGe waveguide. Unlike the conventional gratings of the SOI platform, the SiGe gratings usually have a low coupling efficiency due to the little refractive index difference from the Si substrate. By adding a bottom metal layer on the wafer backside, the coupling efficiency is dramatically improved by approximately 9.4 dB. Moreover, we have designed a two-step apodized grating coupler that achieves a further amelioration of 0.55 dB compared with the uniform design. The influence of the fabrication errors on the coupling efficiency has been analyzed and the proposed grating coupler shows a large tolerance for the deviations. The simulated and measured coupling efficiency of the uniform grating coupler are −1.34 dB and −2.7 dB, respectively. The devised grating coupler paves the way to an efficient fiber-chip coupling for SiGe photonic integration and also provides referential values for designing a grating coupler with a small refractive index difference between the waveguide layer and the substrate.

## Figures and Tables

**Figure 1:** Schematic and cross-section view of the proposed SiGe grating coupler.

**Figure 2:** Coupling efficiency of the grating coupler as a function of etch depth and working wavelength.

**Figure 3:** Coupling efficiency spectra of the proposed grating coupler with and without metal mirror.

**Figure 4:** Simulated (**a**) electrical field component *E_Z_* distribution and (**b**) optical power distribution of the proposed grating coupler with and without the metal mirror.

**Figure 5:** Coupling efficiency spectra of the uniform and apodized grating couplers.

**Figure 6:** Coupling efficiency of the grating coupler as a function of substrate thickness after etching.

**Figure 7:** Coupling efficiency spectra of the grating coupler for different groove width deviations.

**Figure 8:** Coupling efficiency spectra of the grating coupler for different refractive index deviations.

**Figure 9:** The schematic diagram of the fabrication process: (**a**) chip washing (**b**) patterning and etching for waveguide and grating (**c**) deposition of passivation layer (**d**) lithography and deep etching on backside (**e**) metal layer evaporation and lift-off (**f**) the cross section of the whole device.

**Figure 10:** The SEM images of (**a**) the device and (**b**) the zoomed grating. The metalloscope images of (**c**) the chip backside and (**d**) the zoomed bottom metal layer.

**Figure 11:** Test setup diagram.

**Figure 12:** Coupling efficiency of the uniform grating as a function of the wavelength for TE mode.

## Data Availability

The data presented in this study are available on request from the corresponding author.
